# Potential Drug Prediction of Glioblastoma Based on Drug Perturbation-Induced Gene Expression Signatures

This article has been retracted.

**DOI:** 10.1155/2021/6659701

**Published:** 2021-01-25

**Authors:** Bochi Zhu, Xijing Mao, Yuhong Man

**Affiliations:** Department of Neurology, The Second Hospital of Jilin University, Changchun City, Jilin Province, 130041, China

## Abstract

**Objectives:**

Glioblastoma (GBM) is a malignant brain tumor which is the most common and aggressive type of central nervous system cancer, with high morbidity and mortality. Despite lots of systematic studies on the molecular mechanism of glioblastoma, the pathogenesis is still unclear, and effective therapies are relatively rare with surgical resection as the frequently therapeutic intervention. Identification of fundamental molecules and gene networks associated with initiation is critical in glioblastoma drug discovery. In this study, an approach for the prediction of potential drug was developed based on perturbation-induced gene expression signatures.

**Methods:**

We first collected RNA-seq data of 12 pairs of glioblastoma samples and adjacent normal samples from the Gene Expression Omnibus (GEO) database. Differentially expressed genes (DEGs) were identified by DESeq2, and coexpression networks were analyzed with weighted gene correlation network analysis (WGCNA). Furthermore, key driver genes were detected based on the differentially expressed genes and potential chemotherapeutic drugs and targeted drugs were found by correlating the gene expression profiles with drug perturbation database. Finally, RNA-seq data of glioblastoma from The Cancer Genome Atlas (TCGA) dataset was collected as an independent validation dataset to verify our findings.

**Results:**

We identified 1771 significantly DEGs with 446 upregulated genes and 1325 downregulated genes. A total of 24 key drivers were found in the upregulated gene set, and 81 key drivers were found in the downregulated gene set. We screened the Crowd Extracted Expression of Differential Signatures (CREEDS) database to identify drug perturbations that could reverse the key factors of glioblastoma, and a total of 354 drugs were obtained with *p* value < 10^−10^. Finally, 7 drugs that could turn down the expression of upregulated factors and 3 drugs that could reverse the expression of downregulated key factors were selected as potential glioblastoma drugs. In addition, similar results were obtained through the analysis of TCGA as independent dataset.

**Conclusions:**

In this study, we provided a framework of workflow for potential therapeutic drug discovery and predicted 10 potential drugs for glioblastoma therapy.

## 1. Introduction

Glioblastoma (GBM) is a malignant brain tumor which arises from glial cells and is the most common and aggressive type of central nervous system cancer worldwide [1, 2]. To date, surgical resection combined with radiation therapy and chemotherapy is still the frequently therapeutic intervention for GBM [3]. Although some advances in treatment of glioblastoma have been made in recent years, its prognosis is still poor because of its invasive and aggressive behavior. The annual incidence rate of glioblastoma in China is 5-8 per 10 million, and the five-year survival ratio is lower than 5% with a median survival time of 12.6 months. Despite extensive systematic studies on the mechanism of tumorigenesis, metastasis, and recurrence, the underlying mechanism of glioblastoma is still unclear [4] and effective drugs are relatively rare. Therefore, it is crucial to conduct further studies to identify fundamental molecules and gene networks associated with initiation and development, as well as prognosis of GBM, and explore more effective drugs.

High-throughput sequencing has been widely used in cancer research over the past decade, which greatly promotes the understanding of molecular genetics of glioblastoma. TCGA, a landmark cancer genomics program, which contains genomic, epigenomic, transcriptomic, and proteomic data, has also improved our ability to diagnose, treat, and prevent cancer, including glioblastoma. Thus, gene expression profiling has become an objective and important method to classify tumors besides histological classification [5, 6]. A classification of GBM based on platelet-derived growth factor receptor (PDGFR) and the epidermal growth factor receptor (EGFR) has been built [7]. Moreover, molecular subclasses could be utilized to predict prognosis of patients. Methylation status of the O6-methylguanine DNA methyltransferase (MGMT) gene promoter and isocitrate dehydrogenase enzyme 1/2 (IDH1/2) mutation were the prognostic molecules which have been fully confirmed [8, 9]. In addition, IDH mutation status and telomerase reverse transcriptase (TERT) promoter mutation status could enhance prognostic stratification of patients with glioblastoma. Patients with MGMT promoter methylation were more sensitive to temozolomide (TMZ) chemotherapy and had a better prognosis [10]. BRAF (v-raf murine viral oncogene homolog B1) mutations were found in pilocytic astrocytomas and have been proved to be a new therapeutic target for inhibition of the mitogen-activated protein kinase (MAPK) cascade, but its prognostic significance is unknown [11]. Vemurafenib, as a BRAF inhibitor, can have a complete clinical regression of relapsed glioblastoma multiforme [12]. This success has brought great encouragement to the targeted therapies of glioblastoma.

On the other hand, new drug discovery faces many serious challenges, such as a long developing period, substantial cost, high attrition rates, and changing regulatory requirements, which can all contribute to lower yielding for the pharmaceutical industry and a less desirable choice for inventors [13]. Drug repurposing is a strategy for identifying new indication for approved drugs or preclinical compounds. Comparing to developing entirely new drugs from scratch, drug repurposing offers various advantages. The promise of drug repurposing is to accelerate translating the benefits including technology and enhanced knowledge of human disease into therapeutic advances bypassing more time and cost-efficiency. One of the most promising novel methodologies for drug repurposing is computational approaches, such as signature matching, genetic association, and pathway mapping [14, 15]. Omics data can be useful in figuring out not only the mechanism of disease but also pharmacology. By now, the omics technologies can be applied at any molecular levels from genes, RNA, and proteins to metabolites corresponding to genome, transcriptome, and metabolome, respectively. The most widely used omics in drug repurposing is transcriptome and based on which several computational approaches have been proposed [16, 17]. The majority of these strategies were based on transcription profile from cell lines given several large projects based on transcriptome such as LINCS (the library of integrated network-based cellular signatures) [18]. However, there are essential differences between cell lines and tissues, much less to organ and human beings. Therefore, results inferred from omics data based on tissues are more beneficial to drug repurposing.

In this study, the original RNA-seq data with clinical information of glioblastoma samples and adjacent normal samples was downloaded from GEO as testing data. We obtained DEGs by DESeq2, compared gene module changes, and retrieved the potential drugs from CREEDS. Through these studies, we design to understand the mechanism of tumorigenesis and develop systematic research programs for GBM in the future.

## 2. Materials and Methods

### 2.1. Data Collecting

We collected RNA sequencing data of glioblastoma from TCGA and GEO dataset, respectively. 12 pairs of tumor samples and adjacent normal samples were firstly collected from the project ID of GEO-GSE151352 as the testing dataset. For a better verification of our findings, we used an additional data from TCGA as an independent validation dataset which contained 156 tumor samples and 5 normal samples with an expression profile of 60483 genes of each sample.

### 2.2. Differential Gene Expression Analysis between Cancer and Normal Samples

As the input data, the raw read counts were extracted from TCGA dataset or GEO dataset and R package DESeq2 [19] was used for differential gene expression analysis with log2  | fold change | >THRESHOLD_FOLDCHANGE and adjusted *p* value < THRESHOLD_P_ADJ as threshold, where THRESHOLD_FOLDCHANGE and THRESHOLD_P_ADJ are shown in Table 1. The differentially expressed gene analysis was performed between two different conditions. To analyze the biological significance, the biological functions were annotated for the up- or downregulated gene set. Gene Ontology [1, 20] was set as the reference database for the enrichment analysis. R package clusterProfiler [21] was used for the calculations. The R package ggplot2 was used to plot the enriched pathways or functions.

### 2.3. Weighted Gene Correlation Network Analysis and Key Driver Analysis

The genes with ENSEMBL type were converted to gene symbol using map Ids function from the R package clusterProfiler. For WGCNA [22], we used the R package WGCNA for the module discovery. Then, we performed key driver analysis (KDA) as described by Yang et al. [23]. The dynamic neighborhood search (DNS) was applied for KDA. Firstly, we generated a subnetwork NG that is within 2 steps of the nodes in the given gene set. Secondly, for each gene in the NG, DNS was used to find the genes that are within 2 steps of the gene. Thirdly, the hypergeometric test is performed to calculate the *p* value of the enrichment between the gene set from the second step and the input gene set, with the gene set from the first step as the background. The parameters used in the KDA were as follows: with adjusted *p* value < 0.05 for DEG and *p* value for subnet < 0.01 as threshold. We considered key driver genes as hub genes that connected to the up- or downregulated genes.

### 2.4. Drug Prediction

The DEGs and key drivers were applied into the CREEDS to find potential drugs. The dataset could be gained from http://amp.pharm.mssm.edu/creeds.

## 3. Results

### 3.1. Potential Drug Prediction Based on Drug Perturbation-Induced Gene Expression Signatures

We developed a new approach for drug prediction based on drug perturbation-induced gene expression signatures, including DEG analysis, Gene Ontology (GO) enrichment, and key driver analysis, as well as coexpression from WGCNA. Then, the key driver and coexpression genes were combined as key factors of glioblastoma to detect gene and drug perturbation signatures with network pharmacology (Figure 1).

### 3.2. Differentially Expressed Genes Were Gained and Enriched in Different Pathways

We compared the expression profile between the tumor group and the normal group by DEG analysis using DESeq2 [19]. We used the threshold log2 | fold change | >1 and adjusted *p* value < 0.05 for adjusted *p* value. Finally, we got 1771 significantly different expression genes, with 446 upregulated genes (25.2%) and 1325 (74.8%) downregulated genes. The detailed information (log2FC, adjusted *p* value) of 1771 DEGs is listed in Supplementary Table 1. The top 10 upregulated genes and downregulated genes are shown, respectively, in Figure 2(a).

For a better understanding of functions of the upregulated and downregulated genes, we performed GO enrichment analysis on the two gene sets separately, and the threshold of the significance was adjusted *p* value < 0.05. We chose the top ten pathways with the highest proportion of genes for display (Figures 2(b) and 2(c)). The enrichment results showed that the upregulated genes mainly play roles in DNA conformation change, DNA packaging, chromatin assembly or disassembly pathways, extracellular matrix organization, nucleosome organization, and DNA replication-dependent nucleosome assembly or organization, which play an important role in cell differentiation, proliferation, and apoptosis, while the downregulated genes are mainly distributed in signal pathways related to the function of brain nerve cells, such as the modulation of chemical synaptic transmission and the regulation of transsynaptic signaling, which suggests that the occurrence of glioblastoma may affect the function of normal cells.

### 3.3. Weighted Gene Correlation Network Analysis Found Coexpression Modules Perturbed by GBM

To understand the relationship of differentially expressed genes, we attempted to modularize the genes into different modules using WGCNA. The DEG data of the normal group and the GBM group was analyzed separately to observe the synergistic effect of gene expressions under different conditions. The genes with zero expression were removed in all samples; then, the samples with a partially segregated group of the hierarchical clustering results were deleted, and then, weighted gene correlation network analysis was performed. We finally obtained 44 gene modules in the GBM group and 31 gene modules in the normal group. The number of modules and submodules in the GBM group increased, but the coexpression effect of genes decreased, and the signal pathway regulation system tended to be disordered. Then, we randomly selected 400 genes to construct a topological overlapping heat map (Figure 3(a)) and made functional enrichment analysis on the modules (Figures 3(b) and 3(c). As is shown, highly coexpressed genes mainly focused on the mRNA processing, translational initiation, and skeletal system development pathways.

### 3.4. Key Driver Analysis Found Key Drivers Regulating the Gene Sets

We performed key driver analysis of up- and downexpressed genes separately. 24 key drivers were found in the upregulated gene set, and 81 key drivers were found in the downregulated gene set. Top key drivers and corresponding up- or downregulated genes were selected as shown in Figure 4. CAMK2G is short for Calmodulin-Dependent Protein Kinase II Gamma and is one of the hub genes of downregulated genes (Figure 4(b)). Among its related pathways are neuroscience and translation regulation by alpha-1 adrenergic receptors. CDH1 (Cadherin 1) is another hub gene of downregulated genes and participated in regulation of Wnt-mediated beta catenin signaling and target gene transcription (Figure 4(a)). CACNA1G (Calcium Voltage-Gated Channel Subunit Alpha1 G) is a hub gene of upregulated genes that related to regulation of Wnt-mediated beta catenin signaling, target gene transcription, and sweet taste signaling pathways (Figure 4(b)). GLRA3 (Glycine Receptor Alpha 3) is a hub gene of downregulated genes and encodes a member of the ligand-gated ion channel protein family (Figure 4(c)). Its encoded protein is a member of the glycine receptor subfamily. We further discussed the mechanism of these genes in Discussion.

### 3.5. Several Potential Therapeutic Drugs for Glioblastoma Cancer Were Found

We screened the CREEDS to identify drug perturbations that could reverse the DEGs of glioblastoma because the CREEDS dataset contains thousands of single-drug perturbation-induced gene expression signatures collected from GEO. Those gene set-drug pairs with significant *p* value might be valuable to our research. 24 drugs were found when we put upregulated genes and key drivers of upregulated genes into CREEDS with *p* value < 10^−10^ as the threshold. 330 drugs were obtained when downregulated genes and key drivers of downregulated genes were put into CREEDS with the same screening condition. We got 4 drugs that could reverse the expression of downregulated gene and 6 drugs that could reverse the expression of upregulated gene by reviewing the drug profile and previous studies (Table 2). These drugs may be used to treat glioblastoma clinically in the future, such as PD-0332991, which is a selective CDK4/6 inhibitor, and presented outstanding results in phase II clinical trials of estrogen receptor- (ER-) positive HER2-negative breast cancer. It also restricted cell proliferation in preclinical models of hepatocellular carcinoma via promoting a reversible cell cycle arrest [24]. More details of potential drugs were discussed in Discussion.

### 3.6. Independent Dataset Showed Similar Results

The data of GBM from TCGA was used as an independent validation. We obtained 5501 significantly DEGs with 2913 upregulated genes (52.95%) and 2588 (47.05%) downregulated genes. The top 10 pathways through GO enrichment analysis of different expression genes showed similar results on downregulated genes, while there are some major differences between the pathways from upregulated gene enrichment analysis of the two datasets (Figure 5). Based on the different expression genes of TCGA data, 242 and 32 key drivers associated with upregulation and downregulation genes were discovered, separately.

## 4. Discussion

GBM is a highly aggressive malignant brain tumor with a poor prognosis, and effective drugs targeted to GBM are relatively rare. New drug discovery is a long period-consuming and high-cost thing. Therefore, it is quite meaningful to find a new way to discover potential drugs to GBM. In this work, we have built a drug discovery process of glioblastoma based on differentially expressed gene analysis and predicted 10 potential drugs for glioblastoma therapy. RNA sequencing data of tumor samples and adjacent normal samples from patients with glioblastoma were used as input files and potential drug dataset as reference files. Furthermore, we used an independent verification set to prove that this method was feasible.

During the process of analysis, we explored the related signal pathway changes of glioblastoma by enrichment analysis. The upregulated genes mainly play roles in DNA conformation change, DNA packaging, chromatin assembly or disassembly pathways, etc. It is well known that the methylation of DNA can change the conformation of DNA molecules. DNA methyltransferases (DNMT1 and DNMT3b) could regulate and maintain the methylation of promoter and are overexpressed in human cancer. Additionally, it has been reported that DNA methyltransferase mediated transcriptional silencing in malignant glioblastoma [25]. It is suggested that defects of the chromatin architecture underlie GBM pathogenesis [26]. In addition to obtaining the relevant signaling pathways, we also obtained some key genes, such as CDH1, through key driver analyzing. CDH1 is a tumor suppressor gene and a tumor metastasis suppressor gene. It encodes a classical cadherin of the cadherin superfamily and mediates the adhesion between epithelial cells. It is closely related to the occurrence, development, and metastasis of malignant tumors from various epithelial sources. Loss of function of this gene is believed to contribute to the proliferation and metastasis of tumor cells. Mutations in this gene are correlated with gastric, breast, colorectal, and ovarian cancer. CAMK2G could support cancers through activating transcription factors such as AKT1, CREB, and CDK1/2 [27, 28]. Chai et al. reported CAMK2G was related to lung tumor by affecting stem-like traits and suggested these were mediated through NF-*κ*B activation. GO annotations related to this gene include protein homodimerization activity and protein kinase activity [29].

In the potential therapeutic drugs for glioblastoma cancer, 10 drugs were selected after gene-drug screening. Curcumin, a component of turmeric (Curcuma longa), had been proved as safe, affordable, and efficacious drug comparing with chemotherapeutic agents. Curcumin is highly fat dissolving and could induce cell death by activating cell death pathways as well as inducing inhibition of growth/proliferation process [30]. Anaphase-Promoting Complex (APC/C) inhibitors, such as proTAME and apcin, targeted cell cycle proteins for proteasomal-mediated degradation. The targets of APC/C are regulated throughout the cell cycle via two mutually exclusive activator proteins, CDH1 and CDC20 [31]. W-13 is a calmodulin antagonist that could inhibit cell growth and induce cell apoptosis, which may display antitumor effects by binding to CAMK2G protein [32]. DE9A inhibitor plays an important role in cell proliferation, differentiation, and apoptosis via the cGMP signaling pathway [33, 34]. BAY73-6691, a PDE9A inhibitor, can suppress breast cancer cell population growth and induce apoptosis [35]. Kaempferol is a well-known flavonoid, with remarkable bioactivity against various malignant tumors, such as non-small-cell lung cancer (NSCLC), breast cancer, hepatocellular carcinoma (HCC), ovarian cancer (OC), and gastric cancer (GC). However, the detailed mechanisms of kaempferol against numerous cancer types have remained elusive [36]. All-trans-retinoic acid could block the cell cycle, enhance apoptosis, and decrease gastric cancer stem cell (CSC) properties [37]. Drugs with high fat solubility, small molecular weight, and simple chemical structure were believed to penetrate the blood-brain barrier easily. However, the potential therapeutic drugs against glioma with the ability to penetrate the blood-brain barrier are still unknown.

There were still several limitations in our study. The datasets were from public databases, the number of samples was relatively small, and the accuracy of the results needed to be further verified. Furthermore, how many effects of a potential drug in the regulatory network still needs to be studied and verified using experimental data. We will continue to track the progress of glioblastoma research and verify the accuracy of the results.

## 5. Conclusions

In this study, we provided a framework of workflow for potential therapeutic drug discovery through a series of analysis processes and predicted 10 potential drugs for glioblastoma therapy. Whether these drugs are effective in patients with glioblastoma deserves further study.

## Figures and Tables

**Figure 1:** The overall pipeline of potential drug prediction based on drug perturbation-induced gene expression signatures: (a) DEG discovery and key driver analysis; (b) finding modules in gene expression profile by WGCNA; (c) finding drugs targeting glioblastoma by multiple strategies.

**Figure 2:** (a) TOP 10 differentially expressed genes by DESeq2. HS3ST3A1, SYNPO, POSTN, DUSP4, TEAD4, PDIA6, STK17A, SHMT2, METTL7B, and TRIB2 were the top 10 upregulated genes. HBG1, FAM19A2, ANXA3, CORO6, SYT1, PLEKHA1, KCTD16, SNAP25, SAMD12, and AAK1 were the top 10 downregulated genes. (b) The top ten pathways by GO enrichment analysis for upregulated genes and (c) downregulated genes between glioblastoma samples and normal samples. The *x*-axis is the ratio of enriched differential expression genes in the corresponding pathway, and the *y*-axis is the name of the pathway.

**Figure 3:** (a) Topological overlapping heat map by WGCNA. Since there are too many genes to visualize, only 400 randomly selected genes are shown in the topological overlapping heat map. Each module was enriched significantly in specific pathways. GO analysis of module 3 and module 11 are shown in (b) and (c).

**Figure 4:** A subnetwork concerning up-/downregulated genes and key drivers. Purple blocks present upregulated genes, red color accounts for key drivers of upregulated genes, green showed the downregulated genes, and blue illustrated key drivers of downregulated genes.

**Figure 5:** Differentially expressed genes by DESeq2 and enrichment analysis results of TCGA data. (a) The top ten pathways by GO enrichment analysis for downregulated genes and (c) upregulated genes between glioblastoma samples and normal samples. The *x*-axis is the ratio of enriched differential expression genes in the corresponding pathway, and the *y*-axis is the name of the pathway.

**Table 1:** Pipelines and parameters for this work.

Step	Goal	Method	Parameters
1	Differentially expressed genes discovery	DESeq2	For GEO dataset: log2 | fold change | >1, adjusted *p* value < 0.05; for TCGA dataset: log2 | fold change | >2, adjusted *p* value < 0.001.
2	Coexpression analysis	WGCNA	For the T group, the soft power threshold was set to 14. For the N group, the soft power threshold was set to 10.
3	Key driver analysis	Key connector analysis	The protein-protein interaction network was used as the reference network for KDA. Parameters were as follows: --nlayerExpansion for 1, --nlayerSearch for 6, --enrichedNodesPercentCut for -1.
4	Drug discovery	Hypergeometric test	The function phyper was used, and the lower tail parameter was set to true.

**Table 2:** List of potential therapeutic drugs for glioblastoma cancer.

Type	Drug/small molecule	Possible effect	Evidence (DOI)
Up	Curcumin	Curcumin-induced cell death is mediated both by the activation of cell death pathways and by the inhibition of growth/proliferation pathways	10.1208/s12248-009-9128-x
Up	APC/C inhibitors	Target cell cycle proteins for proteasomal-mediated degradation	10.1158/1541-7786.MCR-18-1361
Up	PDE9A inhibitor	Elevates central cGMP levels	10.1158/1535-7163
			10.1111/j.1365-2184.2012.00819.x
Up	W-13	A calmodulin antagonist that inhibits cell growth and induces cell apoptosis	10.3892/or.2019.7022
Down	V-4084	Selectively inhibits MET kinase, affects cell cycle in both tumor and host	10.1186/s12967-015-0667-x
			10.1093/noajnl/vdaa067
Down	Kaempferol	Well-known flavonoid, remarkable bioactivity against various malignant tumors	10.1371/journal.pone.0155264
			10.3892/etm.2019.7886
			10.3892/or.2014.3662
Down	PD-0332991	Selective CDK4/6 inhibitor, outstanding results in phase II clinical trials of estrogen receptor- (ER-) positive HER2-negative breast cancer	10.1136/gutjnl-2016-312268
Down	Dexamethasone	Induces tumor lysis syndrome	10.3747/co.21.1769
			10.1097/00000542-200609000-00042
Down	All-trans-retinoic acid	Blocks the cell cycle, enhances apoptosis, and decreases gastric CSC properties	10.3390/ijms19113388
Down	Erlotinib	Blocks tumor cell growth by targeting EGFR	10.1177/1758834011427927
			10.1056/NEJMoa050753

## Data Availability

The data of glioma in the Gene Expression Omnibus (GEO) dataset was collected from the project ID of GEO-GSE151352. The DEGs and key driver dataset were gained from http://amp.pharm.mssm.edu/creeds.

## Supplementary Materials

Supplementary Materials Supplementary Table 1: the log2FC and adjusted *p* value of 1771 DEGs between GBM and normal samples.
